# Total Saponin of *Dioscorea collettii* Attenuates MSU Crystal-Induced Inflammation by Inhibiting the Activation of the TLR4/NF-*κ*B Signaling Pathway

**DOI:** 10.1155/2021/8728473

**Published:** 2021-10-20

**Authors:** Li Guoying, Li Li, Yang Siyue, Lv Lei, Chen Guangliang

**Affiliations:** ^1^College of Integrative Medicine, Anhui University of Chinese Medicine, Hefei 230012, Anhui, China; ^2^Anhui Province Key Laboratory of Chinese Medicinal Formula, Hefei 230012, Anhui, China; ^3^College of Chemistry, University of California, Berkeley, Berkeley, CA 94720, USA

## Abstract

**Background:**

Rhizomes from *Dioscorea collettii* are extensively used in traditional medicine for the treatment of arthritic diseases, particularly gouty arthritis (GA). This study aims to investigate whether the total saponin of *Dioscorea collettii* (TSD) can attenuate monosodium urate (MSU) crystal-induced inflammatory effects by suppressing the activation of the TLR4/NF-*κ*B signaling pathway *in vivo* and *in vitro*.

**Methods:**

Seventy-two male Wistar rats and THP-1 cells were used in this study. Pathological examination was used to examine the ankle joints of rats. The expression levels of TLR4, NF-*κ*B, MyD88, and IL-1*β* were detected by qRT-PCR, Western blotting, or immunofluorescence.

**Results:**

Compared with those in the normal group, the ankle joints of rats in the model group exhibited significant swelling, synovial tissue hyperplasia, inflammatory cell infiltration, and increased expression of IL-1*β* protein. The joint swelling degree of rats in the TSD high- and medium-dose groups and the colchicine group was significantly decreased, and the histopathology was obviously improved. TSD and colchicine reduced the levels of IL-1*β* and TNF-*α* in synovial fluid. They also decreased the mRNA expression of TLR4, NF-*κ*B, and IL-1*β* in rat joint synovial tissue and the protein expression of TLR4, MyD88, and NF-*κ*B. NF-*κ*B protein expression in both the cytoplasm and nuclei of THP-1 cells showed the opposite trend. Furthermore, immunofluorescence showed that TSD reduced the nuclear translocation of NF-*κ*Bp65 in the model group.

**Conclusion:**

TSD exhibits an anti-inflammatory effect in the MSU-induced inflammation model, and the mechanism may be to reduce the production of cytokines by inhibiting the activation of the TLR4/NF-*κ*B signaling pathway.

## 1. Background

Gout is caused by hyperuricemia (HUA), which leads to the formation and deposition of monosodium urate (MSU) crystals. In recent years, the incidence of HUA and gout has gradually increased. A cohort study of 10039 people in Beijing showed that in people over 50 years old, the prevalence of HUA and gout was 18.1% and 2.8%, respectively [1], and these conditions become serious metabolic diseases that endanger human health. Guidelines recommend a nonsteroidal anti-inflammatory drug (NSAID), colchicine, or corticosteroids. Recognition of the importance of NLRP3 inflammasome activation and bioactive IL-1*β* release in the initiation of gout flares has led to the development of antiIL-1*β* biological therapy for gout flares [2, 3].

Rhizomes from *Dioscorea collettii* contain mainly dioscin, protodioscin, gracillin, and protogracill, and they are commonly used for the treatment of gout and hyperuricemia in traditional Chinese medicine [4, 5]. *D. collettii* and its components have been reported in the literature to have anti-inflammatory, antitumor, antihyperuricemia, immunomodulatory, and lipid-regulating effects [6]. A study showed that TSD can promote the excretion of uric acid and prevent hyperuricemia by regulating the expression of uric acid transporter-1 (URAT1) [7, 8]. TSD also has remarkable anti-inflammatory and analgesic effects, which can inhibit the expression of the cytokine IL-1*β* and obviously improve histopathological lesions in gouty arthritis [9, 10]. Our study demonstrates that TSD can attenuate MSU crystal-induced inflammation by inhibiting the activation of the NALP3 inflammasome and caspase-1 [11, 12]. In addition, TSD has a significant anti-inflammatory effect *in vitro*, reducing the secretion of the inflammatory factors TNF-*α* and IL-1*β* in the THP-1-derived macrophage inflammation model stimulated by MSU [13].

Recent studies [14–16] have found that innate immunity is directly involved in the development of gout, and multiple innate immune cells are involved in recognition and phagocytosis of MSU crystals, activation, and signal transduction of intracellular TLR4/NF-*κ*B and regulation of inflammatory cytokines, such as the production and maturation of IL-1*β*. However, it is not clear whether TSD can interfere with NF-*κ*B by inhibiting the TLR4 signaling pathway *in vivo* and *in vitro*. Therefore, the aim of this study was to determine the protective effects of TSD on MSU-stimulated signaling via TLR4, which in turn affects the MyD88/NF-*κ*B signaling pathway *in vivo* and *in vitro*. The impact of TSDs on the prevention and treatment of AGA may provide an experimental basis for the clinical application of TSDs.

## 2. Materials and Methods

### 2.1. Animals

Seventy-two male Wistar rats aged 6–7 weeks and weighing 250 ± 20 g were purchased from Anhui Medical Laboratory Animal Center [certificate number SCXK (Anhui) 2015–001]. The animals were housed in a room with a temperature of 22 ± 2°C and relative humidity of 55 ± 5% and were given standard chow and water *ad libitum* for the duration of the study. All animal experiments were conducted in accordance with international ethical guidelines and the National Institutes of Health Guide concerning the Care and Use of Laboratory Animals.

### 2.2. Cell Culture

The THP-1 cell line (a human acute monocytic leukemia cell line) was purchased from Shanghai Institute of Cell Biology of the Chinese Academy of Sciences. The cells were cultivated in a humidified incubator at 37°C in a 5% CO_2_ atmosphere with RPMI 1640 supplemented with 10% FBS and 1% antibiotic-antimycotics (100 U/mL penicillin *G* sodium, 100 *μ*g/mL streptomycin sulfate) to a subconfluent state. When the confluence reached 90%, cell passaging was performed. The cell suspension was centrifuged at 800 rpm for 5 min, the supernatant was removed, and complete medium was added for resuspension. The cell suspension was cultured with preheated medium at 37°C at a ratio of 1 : 3. THP-1 cells at generations 4–6 were used in later experiments.

### 2.3. Drugs and Reagents

TSD was extracted by the research group, and the total saponin content was 61.7% [17]. Other reagents were colchicine (purity rate >99%) (Meilunbio Co., Ltd., J1225AS), colchicine tablets (Xishuangbanna Pharmaceutical Co., Ltd.), MSU (Shanghai Yuanye Biotechnology Co., Ltd., S24J9I64369), rat IL-1*β* ELISA kits, rat TNF-*α* ELISA kits (Wuhan Boster Bios Co., Lot : EK0393 and EK0526, respectively), TLR4 antibody, MyD88 antibody, NF-*κ*B antibody, *β*-actin antibody (Abcam, ab13556, ab2064, ab16502, and ab8227, respectively), Lamin B antibody (Affinity, AF5161), PCNA antibody (Abbkine, A01040), GAPDH antibody (Servicebio, GB12002), HRP-labeled goat antirabbit IgG, HRP-labeled goat antimouse IgG (Abbkine A21020 and A21010), and ECL chemiluminescence kit (Thermo 32109).

### 2.4. Main Instruments

The instruments used included a multiscan MK3 microplate reader (Thermo, USA), CKX-41 inverted optical microscope (Olympus, Japan), TB-718 biological tissue embedding machine (Hubei Taiwei Electronics Company), NOVA ultrathin slicer (LKB Company), electrophoresis instrument (Bio-Rad, USA), Flour Chem *M* Gel Imaging system (Protein Simple, USA), and Quantstudio Multiple Real-Time PCR System (Life Technologies, USA).

### 2.5. Grouping and Modeling

After one week of adaptive feeding in rats, the rats were randomly divided into the normal group; model group; high-, middle-, and low-dose TSD (300, 100, 30 mg/kg/d) groups; and the colchicine group (0.5 mg/kg/d). There were 12 rats in each group. Rats received intragastric administration of drug 2 times per day for 5 consecutive days. On the third day after administration, 0.2 mL of MSU suspension (25 mg/kg) was injected into the joint cavity on the dorsal side of the right ankle joints [18]. The normal group was injected with the same volume of normal saline as that of MSU.

THP-1 cells were divided into a normal group; a model group; high-, middle-, and low-dose TSD (10, 3, 1 *μ*g/mL) groups; and a colchicine group (0.2 *μ*g/mL). After 12 h of drug pretreatment, all groups except the normal group were stimulated with 400 *μ*g/mL MSU for 6 h to establish a model of cell inflammation.

### 2.6. Measurement of Joint Swelling

Referring to the literature method [19], the circumference of the same part of the right ankle joint was measured with an inelastic tapeline at 0, 6, 12, 24, and 48 h before and after the modeling. The measurement was repeated 3 times, and the average was taken. Joint swelling degree was referred to as joint circumference after modeling-joint circumference before modeling.

### 2.7. Enzyme-Linked Immunosorbent Assays (ELISAs)

Rats were anesthetized with 0.3% pentobarbital sodium and sacrificed at the designated time. The paw was cutoff, and an incision was made at 0.5 cm from the right ankle joint. The skin was peeled off in a small beaker containing 5 mL of normal saline. The surrounding tissue was cut, and the liquid containing the tissue was moved into a centrifuge tube, shaken for 10 min, soaked for 1 h, and then centrifuged at 4°C and 25000 rpm for 10 min. The supernatant was taken to detect relevant indicators. The contents of IL-1*β* and TNF-*α* were determined by strictly following the instructions of the double-antibody Sandwich ELISA kit.

### 2.8. Histopathological Examination (HE)

The rats were sacrificed 48 h after modeling, and the ankle joint and surrounding soft tissue were collected. After fixation for 1 week with 4% paraformaldehyde, the tissues were decalcified in 8% hydrochloric acid-formaldehyde decalcification solution, dehydrated in gradient alcohol solutions, embedded in paraffin, and longitudinally sectioned at 5 *μ*m. HE staining and filming were subsequently performed.

#### 2.8.1. Immunohistochemistry for the Detection of IL-1*β* Expression in Rat Synovial Tissue

The rats were sacrificed in the same way as described above. After fixation of the ankle joints in 4% paraformaldehyde for 24 h, the joint tissues were decalcified in EDTA decalcification solution for 2 months. The decalcifying solution was changed once per week until the ankle joint became soft and could be cut with a knife. The ankle joints underwent gradient alcohol dehydration, conventional paraffin embedding, longitudinal sectioning at 5 *μ*m, dewaxing hydration, antigen retrieval, and blocking with 3% H_2_O_2_. After incubation with an IL-1*β* antibody, the sections were stained with DAB, counterstained with hematoxylin, and dehydrated in ethanol. Xylene was added dropwise to clear the tissue, and the film was sealed with neutral resin and observed under a microscope.

#### 2.8.2. Detection of TLR4, NF-*κ*B, and IL-1*β* mRNA Expression in Rat Synovial Tissue by RT-qPCR

Total RNA was extracted from joint synovial tissue with a TRIzol kit, and the integrity of the RNA was verified by denaturing agarose gel electrophoresis. The target gene cDNA fragment was amplified by using Unvi Company's QuantiNova Rev. The qPCR primer sequences were designed by Primer-BLAST according to an NCBI gene pool query of the gene mRNA sequences, and primers specific for the TLR4, NF-*κ*B, and IL-1*β* genes were synthesized by Shanghai Sangon Co., Ltd. (Shanghai, China). The primer sequences are provided in Table 1. After amplification, *β*-actin was used as the internal reference gene, and ^Δ^C_t_ and ^ΔΔ^*C*_*t*_ were calculated according to the following formula: ^Δ^*C*_*t*_ = *C*_t_ target gene-Ct reference gene; ^ΔΔ^*C*_*t*_ = (*C*_t_ experimental group target gene - *C*_t_ experimental group internal reference gene)-(*C*_t_ normal group target gene – *C*_t_ normal group internal reference gene). All samples were run in triplicate, and gene expression levels were quantified using the 2^−ΔΔCT^ method as previously described [20].

Detection of TLR4/NF-*κ*B signaling pathway-related protein expression in rat synovial tissue and NF-*κ*B in both the cytoplasm and nuclei of THP-1 cells by Western blot assay.

All proteins were extracted on ice to maintain the stability of the proteins. The synovial membrane was placed in a 1-mL Eppendorf (EP) tube, and RIPA lysate containing 1 mM PMSF was directly added. The pipette was repeatedly triturated to completely lyse the synovial tissue, which was then centrifuged at 4°C and 12000 rpm for 5 min to collect the protein sample for quantification by the BCA method. To detect the expression levels of NF-*κ*B p65 in the nucleus and cytoplasm, the proteins were extracted separately via Nuclear-Cytosol Extraction Kits (Applygen Technologies Inc., Beijing, China). Western blot analysis was used to measure the expression of TLR4, MyD88, and NF-*κ*B p65 (cytoplasm and nucleus). ECL hypersensitive luminescence solution was used for chemiluminescence, and the Protein Simple Fluor Chem *M* ultrasensitive automatic multicolor fluorescence/chemiluminescence imaging system was used for exposure.

#### 2.8.3. Detection of NF-*κ*Bp65 in MSU-Induced THP-1 Cells by Immunofluorescence Assay

THP-1 cells were seeded into 6-well plates with glass coverslips (approximately 2 × 10^4^ cells per well). After adherence, six different groups of cells were subjected to immunofluorescence staining. In detail, the cells were washed three times with PBS and then fixed in 4% phosphate-buffered paraformaldehyde for 30 min. Next, the cells underwent permeabilization with 0.1% Triton X-100 for 20 min, were incubated with fetal bovine serum (FBS) for 1 h, and were subsequently incubated with antiNF-*κ*B p65 polyclonal antibodies (1 : 500) overnight at 4°C. After being washed with PBS three times for 5 min, the cells were incubated with goat antirabbit IgG (*H* + *L*) (1 : 200) for 2 h, the antibody solution was discarded, and the cells were washed with PBS. Finally, the blue and green fluorescence of the cells on the coverslip was observed under an OLYMPUS IX71 inverted phase contrast fluorescence microscope, and pictures were taken. NF-*κ*Bp65 fluoresced green, and DAPI, which stained cell nuclei, fluoresced blue. ImageJ was used to superimpose the images to assess the nuclear translocation of NF-*κ*Bp65.

### 2.9. Statistical Analysis

Data processing was performed by SPSS 23.0 and GraphPad Prism version 7.0. All the data are expressed as the mean ± standard error, and Student's *t*-test was used to compare differences between two groups. One-way ANOVA was applied to assess differences between multiple groups, and multiple comparisons within the groups were performed. A value of *P* < 0.05 was considered statistically significant.

## 3. Results

### 3.1. Effect of TSD on Joint Swelling in GA Rats

Compared with those in the normal group, the ankle joint of rats in the model group showed significant swelling at 6 h after injection, and the swelling peaked at 24 h to 48 h. Compared with the model group, the degree of joint swelling in the colchicine group and the high- and middle-dose TSD groups at 6–48 h was significantly decreased, but there was no significant difference in the degree of joint swelling in the low-dose group (Figure 1).

### 3.2. Effect of TSD on TNF-*α* and IL-1*β* in Joint Synovial Fluid in GA Rats

Compared with those in the normal group, the levels of TNF-*α* and IL-1*β* in the joint synovial fluid in the model group were significantly increased. Compared with those in the model group, the levels of TNF-*α* and IL-1*β* in the colchicine group and the high- and middle-dose TSD groups were significantly decreased (*P* < 0.01) (Figure 2).

### 3.3. Effect of TSD on the Pathomorphology of Ankle Synovial Tissue in GA Rats

In the normal group, the synovial tissue structure of the ankle joint was clear, and there was no or very little inflammatory cell infiltration. The inflammatory response of the synovial tissue in the model group was obvious. The synovial tissue was disordered, and cell proliferation was clearly visible. The cells were congested, showing edema and partial synovial tissue necrosis, and this change was accompanied by a large amount of inflammatory cell infiltration; synovial tissue cells in the colchicine group; and the high-dose TSD group was basically normal or slightly hyperplastic, showing mild congestion and edema, and a small amount of inflammatory cell infiltration was observed. The synovial tissue cells in the middle- and low-dose TSD groups had more hyperplasia, and the synovial cells and surrounding tissues had different degrees of congestion, edema, and inflammatory cell infiltration (Figure 3).

### 3.4. Effect of TSD on the Expression of IL-1*β* in Rat Synovial Tissues

Compared with the normal group, the expression of IL-1*β* in the model group was significantly increased (*P* < 0.01). Compared with the model group, the expression of IL-1*β* was significantly decreased in the colchicine group and the high- and middle-dose TSD groups (*P* < 0.01) (Figure 4).

### 3.5. Effect of TSD on the mRNA Expression of TLR4, NF-*κ*B, and IL-1*β* in the Synovial Tissues of GA Rats

Compared with the normal group, TLR4, NF-Κb, and IL-1*β* mRNA expression in the model group was significantly increased (*P* < 0.01). Similar to colchicine treatment, the administration of TSD significantly inhibited the mRNA expression of TLR4, NF-*κ*B, and IL-1*β* in the synovial tissues of MSU-induced GA rats in a dose-dependent manner (Figure 5).

### 3.6. Effect of TSD on the Expression of TLR4, MyD88, and NF-*κ*Bp65 in the Synovial Tissues of GA Rats

Western blotting and semiquantitative statistics showed that compared with the normal group, TLR4, MyD88, and NF-*κ*Bp65 levels in the model group were significantly increased (*P* < 0.01). TSD significantly reduced the levels of these proteins in a dose-dependent manner. The levels of TLR4, MyD88, and NF-*κ*Bp65 were significantly decreased in the colchicine group (Figure 6).

### 3.7. Effect of TSD on the Expression of NF-*κ*B in Both the Cytoplasm and Nuclei of THP-1 Cells

Compared with the normal group, NF-*κ*B expression was significantly decreased in the cytoplasm in the model group, and the opposite trend was observed in the nucleus (*P* < 0.01). In addition, TSD increased the expression of NF-*κ*B in the cytoplasm in a dose-dependent manner while decreasing NF-*κ*B expression in the nuclei, which was consistent with the *in vivo* results (Figure 7).

### 3.8. Effect of TSD on the Nuclear Activation of NF-*κ*Bp65 in THP-1 Cells

The green fluorescence indicated NF-*κ*Bp65 staining, and the blue fluorescence indicated DAPI staining of the cell nucleus. In the normal group, NF-*κ*Bp65 was expressed mainly in the cytoplasm, the blue cell nuclei had clear boundaries, and the green fluorescence in the nuclei of the model group gradually increased. ImageJ was used to superimpose the images to assess the nuclear translocation of NF-*κ*Bp65. The nucleus showed clear turquoise fluorescence, indicating that NF-*κ*Bp65 was located in the nuclei. The degree of superimposition was decreased in the TSD and colchicine groups, indicating that TSD and colchicine inhibited the translocation of NF-*κ*B from the cytoplasm to the nuclei. That is, TSD and colchicine inhibited the activation of NF-*κ*B, thereby reducing the synthesis and activation of the inflammatory factor IL-1*β* (Figure 8).

## 4. Discussion

Although gout is an ancient disease, it is not understood at the molecular and cellular levels. The TLR/MyD88/NF-*κ*B receptor signaling pathway synergizes with the NALP3 inflammasome to activate IL-1*β*, which plays a key role in gout inflammation caused by MSU crystals. After hyperuricemia of blood uric acid, MSU crystals are deposited in joints and soft tissues, which are recognized by pattern recognition receptors (such as TLRs and NODs), and various innate immune cells participate in the recognition and engulfment of MSU crystals. Activated Toll-like receptors activate NF-*κ*B via the cytoplasmic adaptor protein MyD88 and initiate transcription and expression of the precursor IL-1*β* gene, which is cleaved into mature IL-1*β* and secreted extracellularly, causing neutrophil recruitment and the release of more inflammatory mediators, producing an inflammatory cascade amplification reaction that induces acute gouty arthritis episodes [21–23]. Briefly, the signaling pathway involved in Toll-like receptors is responsible for the production of precursor IL-1*β*, while the NALP3 inflammasome is responsible for the cleavage and activation of precursor IL-1*β*, forming active IL-1*β*. The IL-1 receptor antagonists anakinra, rilonacept, and canakinumab can effectively alleviate the symptoms of acute gout and have become the fourth class of drugs for the treatment of acute gout [24].

Clinically, the presence of uric acid crystals in the joint fluid, bursa, or tophi can be directly diagnosed as gout [25]. Injecting MSU crystals into the joint cavity results in a model of acute gouty arthritis, and its pathological findings are very similar to clinical findings. In this experiment, the acute joint inflammatory model was replicated by the injection of MSU into the ankle joint of the rats. The degree of joint swelling was significantly increased after the model was established, and the hind limbs were lifted off the ground. Pathological observation of the affected ankle joints showed that synovial tissue cells proliferated and that partial necrosis was accompanied by a large amount of inflammatory cell infiltration, congestion, and edema. Compared with the model group, the joint swelling degree in the high- and medium-dose TSD groups and the colchicine group was significantly decreased between 6 and 48 h. The synovial tissue cells were basically normal or slightly hyperplastic, and mild hyperemic edema was observed in the cartilage tissue around the ankle joint. A small amount of infiltration or infiltration of inflammatory cells was not obvious. The results showed that TSD had significant preventive effects on acute gouty arthritis in rats, and its effect was similar to the effect of colchicine.

IL-1*β* is a key inflammatory factor that mediates gouty arthritis. IL-1*β* activates the IL-1 signaling pathway and MyD88-dependent NF-*κ*B signaling pathway by binding to the IL-1 receptor, which leads to the transcription of a large number of proinflammatory factors, such as IL-1, TNF-*α*, and IL-8, and produces an inflammatory cascade amplification effect [26]. The expression of IL-1*β* and TNF-*α* in the joint synovial fluid of MSU-induced GA rats in the model group was significantly increased, suggesting that inflammatory factors such as IL-1*β* and TNF-*α* play an important role in acute episodes of gout. Compared with the model group, IL-1*β* expression was significantly decreased in the swollen joint synovial fluid of the high- and medium-dose TSD groups and the colchicine group, suggesting that high- and medium-dose TSD could inhibit the expression of inflammatory factors.

NF-*κ*B is a common transcription factor activated by inflammatory factors, growth factors, or chemokines. Bound to I*κ*B, inactive NF-*κ*B stays in the cytoplasm; when I*κ*B is phosphorylated by IKK*α*/*β* and subsequently degraded, unbound NF-*κ*B is released and translocates to the nucleus, initiating mRNA transcription of downstream genes. Therefore, whether the major subunit p65 of NF-*κ*B is transferred to the nucleus is the main basis for judging NF-*κ*B activation. Compared with the model group, the translocation of NF-*κ*B from the cytoplasm into the nucleus was inhibited in the TSD and colchicine groups, indicating that inflammation was alleviated to some extent.

The TLR/MyD88/NF-*κ*B receptor signaling pathway plays an important role in acute gout. TLRs belong to a family of pattern recognition receptors and can recognize pathogen-associated molecular patterns (PAMPs). TLR recognizes the corresponding ligands, binds to these ligands, and transmits signals via the MyD88-dependent pathway through its cytoplasmic region Toll/interleukin-1 receptor (IL-1R) homology domain (Toll/IL-1R domain, TIR), which combines with the MyD88 C-terminal TIR to form a complex. Furthermore, NF-*κ*B is activated to induce the expression of inflammatory cytokines such as IL-1, TNF-*α*, and adhesion molecules to promote inflammation [21, 27]. The expression of TLR4, MyD88, NF-*κ*B, and IL-1*β* in the synovial tissue of the model group was significantly upregulated, indicating that the TLR/MyD88/NF-*κ*B receptor signaling pathway was involved in the development of acute gouty arthritis in rats. Compared with the model group, the protein expression of TLR4, MyD88, and NF-*κ*B was significantly decreased in the high- and medium-dose TSD groups and the colchicine group, indicating that the effect of TSD against gouty arthritis might occur through the suppression of the TLR/MyD88/NF-*κ*B receptor signaling pathway and the activation of inflammatory factors, the role of which was similar to the role of colchicine.

## 5. Conclusions

In summary, TSD exhibits an anti-inflammatory effect in the MSU-induced inflammation model, and the mechanism may be to suppress the activation of the TLR4/NF-*κ*B signaling pathway and reduce the production of cytokines.

## Figures and Tables

**Figure 1:** Effect of TSD on joint swelling in MSU-induced GA rats at 48 h (scale bar = 1 cm, *n* = 12). Compared with the normal group, ^##^*P* < 0.01; compared with the model group, ^*∗∗*^*P* < 0.01, ^*∗*^*P* < 0.05.

**Figure 2:** Effect of TSD on the levels of IL-1*β* and TNF-*α* in MSU-induced GA rats (*n* = 6). Compared with the normal group, ^##^*P* < 0.01; compared with the model group, ^*∗∗*^*P* < 0.01, ^*∗*^*P* < 0.05.

**Figure 3:** Effect of TSD on the pathological morphology of synovial tissue in MSU-induced rats (scale bar = 0.1 mm).

**Figure 4:** Effect of TSD on the expression of IL-1*β* in rat synovial tissue (scale bar = 0.1 mm).

**Figure 5:** Effect of TSD on the expression of TLR4, NF-*κ*B, and IL-1*β* mRNA in the MSU-induced synovial tissue of GA rats (*n* = 6). Compared with the normal group, ^##^*P* < 0.01; compared with the model group, ^*∗∗*^*P* < 0.01.

**Figure 6:** Effect of TSD on the expression of TLR4, MyD88, and NF-*κ*Bp65 in the synovial tissue of GA rats (*n* = 6). Compared with the normal group, ^##^*P* < 0.01; compared with the model group, ^*∗∗*^*P* < 0.01 and ^∗^*P* < 0.05.

**Figure 7:** Effect of TSD on the expression of NF-*κ*B in both the cytoplasm and nuclei of THP-1 cells (*n* = 3). Compared with the normal group,^##^*P* < 0.01; compared with the model group, ^*∗∗*^*P* < 0.01and ^∗^*P* < 0.05.

**Figure 8:** Effect of TSD on the nuclear transcriptional activation of NF-*κ*Bp65 in THP-1 cells was detected by immunofluorescence (scale bar = 50 *μ*m).

**Table 1:** Primer sequence of RT-qPCR.

Primers	Genbank accession	Primer sequences (5' ⟶ 3′)
TLR4	NM_019178.1	ACATAGCAGATGTTCCTAGGCA GCCAACTGACCAAAGCTGATAT
NF-*κ*B	NM_001276711.1	ACGGGAGGGGAAGAAATCTATC AATGGCAAACTGTCTGTGAACA
IL-1*β*	NM_031512.2	GACCTGCTAGTGTGTGATGTTC CATTGAGGTGGAGAGCTTTCAG
*β*-actin	NM_031144.3	CTTCCTTCCTGGGTATGGAATC CTGTGTTGGCATAGAGGTCTT

## Data Availability

The datasets analyzed during the current study are available from the corresponding author upon reasonable request.
